This article has been retracted.

# Effect of rosuvastatin on fasting and postprandial endothelial biomarker levels and microvascular reactivity in patients with type 2 diabetes and dyslipidemia: a preliminary report

**DOI:** 10.1186/s12933-017-0629-0

**Published:** 2017-11-09

**Authors:** Kyoung Min Kim, Kyong Yeun Jung, Han Mi Yun, Seo Young Lee, Tae Jung Oh, Hak Chul Jang, Soo Lim

**Affiliations:** 1 Department of Internal Medicine, Seoul National University College of Medicine and Seoul National University Bundang Hospital, 82 Gumi-ro 173beon-gil, Bundang-gu, Seongnam, 463-707 South Korea; 2 Department of Internal Medicine, Eulji General Hospital, Seoul, South Korea; 3 Physiologic Diagnostic Laboratory, Vascular Laboratory, Seoul National University Bundang Hospital, Seongnam, South Korea

**Keywords:** Endothelial function, Microvascular reactivity, Paraoxonase 1, Asymmetric dimethylarginine, Rosuvastatin, Type 2 diabetes

## Abstract

**Background:**

The cardiovascular benefits of statins have been proven, but their effect on circulation in small vessels has not been examined fully. We investigated the effect of 20 mg rosuvastatin on biomarkers, including paraoxonase-1 (PON-1) and asymmetric dimethylarginine (ADMA), and on microvascular reactivity.

**Method:**

We enrolled 20 dyslipidemic patients with type 2 diabetes and 20 age- and body mass index (BMI)-matched healthy controls. Rosuvastatin (20 mg/day) was given to the patient group for 12 weeks. Biochemical parameters, including PON-1 and ADMA, were compared between the patient and control groups, and before and after rosuvastatin treatment in the patient group. Fasting and 2 h postprandial levels of PON-1 and ADMA after mixed-meal challenge were also compared. Microvascular reactivity in a peripheral artery was examined using laser Doppler flowmetry.

**Results:**

The respective mean ± standard deviation of age and BMI were 50.1 ± 3.8 year and 25.8 ± 3.7 kg/m^2^ in the patients and 50.2 ± 3.2 year and 25.4 ± 3.4 kg/m^2^ in the controls. The patient group had worse profiles of cardiometabolic biomarkers, including PON-1 and ADMA, than the controls. In the patients treated with 20 mg rosuvastatin, low-density lipoprotein (LDL)-cholesterol decreased from 147.2 ± 26.5 to 68.3 ± 24.5 mg/dL and high-density lipoprotein (HDL)-cholesterol increased from 42.4 ± 5.2 to 44.7 ± 6.2 mg/dL (both *P* < 0.05). Both fasting and 2 h postprandial levels of PON-1 increased and those of ADMA decreased after treatment with rosuvastatin for 12 weeks. The changes in postprandial levels of both biomarkers were greater than those after fasting. Microcirculation assessed as reactive hyperemia in the patients after an ischemic challenge increased significantly from 335.3 ± 123.4 to 402.7 ± 133.4% after rosuvastatin treatment. The postprandial changes in the biomarkers were significantly associated with improvement of microvascular reactivity.

**Conclusions:**

Rosuvastatin treatment for 12 weeks improved microvascular reactivity with concomitant beneficial changes in the postprandial levels of PON-1 and ADMA. These results suggest that rosuvastatin improves the postprandial cardiometabolic milieu in type 2 diabetes.

*Trial registration* ClinicalTrials.gov: NCT02185963 (July 7, 2014)

**Electronic supplementary material:**

The online version of this article (10.1186/s12933-017-0629-0) contains supplementary material, which is available to authorized users.

## Introduction

The cardiovascular benefits of statin treatment have been proven in patients with type 2 diabetes (T2D) [1]. In the Collaborative Atorvastatin Diabetes Study, atorvastatin (10 mg/day) was found to be efficacious in reducing the risk of cardiovascular events in patients with T2D, even those without high levels of low-density lipoprotein (LDL)-cholesterol [2]. In the “Justification for the Use of Statins in Prevention: An Intervention Trial Evaluating Rosuvastatin” trial, treatment with 20 mg rosuvastatin reduced major cardiovascular events in 17,802 healthy individuals with relatively low levels of LDL-cholesterol for up to 5 years [3].

However, studies that have investigated the effects of statins on circulation in small vessels are limited. A recent study reported that treatment with 20 mg pravastatin for 6 months improved fasting and postprandial endothelial dysfunction as assessed by forearm blood flow during post-ischemic reactive hyperemia in patients with angina [4]. In a study of patients undergoing primary coronary intervention, treatment of 40 mg atorvastatin before and after the procedure reduced circulating levels of endothelin-1, a marker of endothelial dysfunction [5].

Several biomarkers are directly related to endothelial function or microcirculation. Among them, asymmetric dimethylarginine (ADMA) and paraoxonase-1 (PON-1) have drawn attention. ADMA is a dimethylarginine structurally related to l-arginine. It is considered a key regulator of vascular tone because it inhibits the production of nitric oxide (NO). A study using metabolomics has identified ADMA as a new biomarker of chronic kidney disease [6]. High ADMA level leads to a decrease in NO production, indicating its association with endothelial dysfunction [7]. Cross-sectional studies have found that ADMA levels are elevated in persons with T2D and macrovascular disease [8, 9]. Moreover, ADMA is an independent risk factor for cardiovascular disease and mortality in a wide spectrum of populations [10, 11].

PON-1 is an enzyme associated with high-density lipoprotein (HDL), and several studies have shown that PON-1 has antioxidant and antiatherosclerotic effects. This enzyme hydrolyzes aromatic carboxylic acid esters, organophosphates, and oxidized phospholipids. Thus, PON-1 protects against lipid oxidation, leading to a decrease in oxidized lipoprotein production [12, 13]. Decreased PON-1 activity is associated with accelerated atherosclerosis [14]. A meta-analysis suggested that statin therapy is associated with a significant elevation of PON-1 activity [15].

Skin microvascular reactivity, as measured noninvasively by laser Doppler flowmetry, is a parameter that can be used to assess the responsiveness of microcirculation to occlusion or temperature [16]. Microvascular reactivity is attenuated in insulin-resistant conditions, and is an independent marker of future cardiovascular events in patients with T2D. Therefore, it has been recently adopted to assess endothelial function at an early stage [17, 18].

Postprandial lipid profiles are thought to be important in vascular health. The cardiovascular milieu around the vascular endothelium is aggravated particularly after a high-fat meal. A recent study showed that a high-fat diet increased NO consumption in the circulation [19]. Given that the removal of the lipids from the plasma decelerates NO consumption, statin treatment might be able to improve an unfavorable endothelial milieu after food intake. However, to our knowledge, there is no study that has investigated the effect of a statin on postprandial levels of vascular biomarkers such ADMA or PON-1 and their association with circulation in small vessels. Given that most people spend about half of each day in postprandial status, it would be intriguing to know whether high-intensity statin treatment may influence microcirculation, and, moreover, differently affect levels of biomarkers in fasting and postprandial status.

The purpose of this study was to investigate the effect of rosuvastatin biomarkers related to endothelial function, focusing on ADMA and PON-1, and microvascular reactivity in patients with T2D. We also assessed whether changes in fasting and postprandial levels of ADMA or PON-1 are associated with microvascular reactivity.

## Methods

### Patients and design

We recruited 20 patients with T2D and dyslipidemia and 20 age- and body-mass index (BMI)-matched healthy controls. Inclusion criteria for the patients group were individual with age ≥ 20 year, T2D with HbA1c ≥ 6.5%, LDL-cholesterol level ≥ 100 mg/dL, and HDL-cholesterol level < 40 mg/dL in men and < 50 mg/dL in women. Exclusion criteria were contraindications to statins, a statin medication history within 12 weeks of study enrollment, and aspartate or alanine aminotransferase (AST or ALT) levels > 3 times above the upper normal range. For the healthy control group, individuals who had normal glucose and lipid profiles without cardiovascular risk and were ± 3 years of the age and ± 2 kg/m^2^ of the BMI of the patient participants were selected.

First, we compared biochemical parameters and microcirculation between the patients and healthy controls. In addition to lipid and glucose metabolism parameters, vascular biomarkers such as ADMA and PON-1 levels were measured at fasting and in the 2 h postprandial condition after the mixed-meal challenge in both patients and controls. Second, in the patient group, we investigated changes in microcirculation and fasting and postprandial levels of ADMA and PON-1 between baseline and after 12 weeks of treatment with 20 mg rosuvastatin daily.

This study was approved by the Institutional Review Board of Seoul National University Bundang Hospital (SNUBH) (IRB no. B-1403-241-008) and complied with the principles of the Declaration of Helsinki and its contemporary amendments. This study was registered at ClinicalTrials.gov: NCT02185963. All participants provided their written informed consent to participate before enrollment in this study.

### Anthropometric parameters

Height and body weight were measured by standard methods with the participants in light clothing. BMI was calculated as body weight (in kg) divided by the square of the height (in m).

### Mixed-meal test

We used a commercialized formula for the standardized meal test (New Care, Daesang, Seoul, South Korea). A can of New Care contains 200 kcal, 28 g of carbohydrates, 8 g of protein, 7 g of fat, and 180 mg of sodium. Detailed information of the individual nutrient content is shown in Additional file 1: Table S1. Two and a half cans of New Care (500 kcal in total) were given to each patient participant who had been in a fasting state for 10 h. Blood samples were obtained at fasting and 2 h postprandially.

### Biochemical parameters

After 10 h of overnight fasting, venous blood samples were taken for biochemical assays at baseline and after rosuvastatin treatment. The serum levels of total cholesterol, triglycerides, HDL-cholesterol, and LDL-cholesterol were measured using a Hitachi 747 Clinical Chemistry Analyzer (Hitachi, Tokyo, Japan). Aspartate aminotransferase/alanine aminotransferase (AST/ALT) and creatinine were measured using an Architect Ci8200 analyzer (Abbott Laboratories, Abbott Park, IL, USA).

Plasma glucose concentration was measured using a glucose oxidase method (747 Clinical Chemistry Analyzer; Hitachi). Glycated hemoglobin (HbA1c) levels were measured using a Bio-Rad Variant II Turbo HPLC Analyzer (Bio-Rad, Hercules, CA, USA) in the National Glycohemoglobin Standardization Program level II certified laboratory at SNUBH. Fasting insulin levels were measured by radioimmunoassay (Linco, St. Louis, MO, USA). The homeostasis model assessments of insulin resistance (HOMA-IR) and β-cell function (HOMA-β) were calculated [20]. High-sensitivity C-reactive protein (hsCRP) levels were measured with a high-sensitivity automated immunoturbidimetric method (CRP II Latex 3; Denka Seiken, Tokyo, Japan).

### Measurement of specific biomarkers related to endothelial function

Blood was centrifuged immediately after collection from each participant, and the plasma was frozen and stored at − 80 °C. The maximal storage time of the plasma samples before analysis of biomarkers was 6 months.

PON-1 activity was measured in serum using commercial enzyme-linked immunosorbent assay kits according to the manufacturer’s instructions (VersaMax; Molecular Devices, Sunnyvale, CA, USA) [21]. The intra- and interassay coefficients of variation for the assays were 4.2 and 6.1%, respectively.

Plasma concentrations of ADMA were determined by high-performance liquid chromatography/mass spectrometry simultaneously with fluorescence detection (LC–MS/MS, Agilent Technologies, Santa Clara, CA, USA) as previously described [22], using modified chromatographic separation conditions [23]. For ADMA, the intra- and interassay coefficients of variation were < 2.1 and < 4.2%, respectively.

### Assessment of microvascular reactivity in small vessels

Vascular health was assessed by microcirculation using a laser Doppler system in a fasting state in both controls and patients, and was repeated after 12 weeks of rosuvastatin treatment only in the patient group. To measure microvascular flow, a Laser Doppler perfusion monitor system (PeriFlux System 5000, Perimed, Stockholm, Sweden) was used [18]. This system operates with two laser diodes that emit light with a wavelength of 780 nm. The Laser Doppler probe was applied at the dorsum of the hand, avoiding any underlying bony structures or large vessels. Mean blood flow was measured over 1 min while patients were resting. Postocclusive reactive hyperemia was assessed during the examination by a 5-min occlusion of the upper limb, which was performed using a cuff placed on the upper arm. The pressure of the cuff was 50 mmHg higher than the systolic pressure measured on the upper arm. The maximal flow within 5 min after release of the cuff was recorded.

### Statistical analysis

Data are given as the mean ± standard deviation (SD). Baseline characteristics were compared between the patient and control groups using a Student *t* or Mann–Whitney U test. A paired *t* test or Wilcoxon signed-rank test was used to compare various factors before and after statin treatment. The Pearson correlation coefficient was analyzed to evaluate the association between levels of biomarkers and microcirculation. We considered *P* < 0.05 to be significant. Statistical analyses were performed using SPSS Statistics for Windows (version 20.0, IBM Corp, Armonk, NY, USA).

## Results

### Comparison of biochemical parameters between patients with diabetes and healthy controls

Clinical and biochemical characteristics in the 20 dyslipidemic patients with T2D and 20 age- and BMI-matched healthy controls are presented in Table 1. They were generally middle aged and moderately overweight. Among the patients with T2D, five were managed with lifestyle modification alone, eight with metformin alone, and seven with metformin plus other hypoglycemic agents.

**Table 1:** Baseline characteristics of patients with type 2 diabetes and dyslipidemia and the healthy controls

	DM patients	Healthy controls	P
Age (year)	52.3 ± 9.9	52.0 ± 7.7	NS
Height (cm)	164.2 ± 9.4	165.4 ± 9.6	NS
Weight (kg)	66.8 ± 12.4	66.7 ± 11.0	NS
BMI (kg/m^2^)	24.6 ± 2.8	24.2 ± 1.9	NS
Total cholesterol (mg/dL)	233.4 ± 36.5	183.8 ± 20.4	< 0.001
Triglycerides (mg/dL)	230.5 ± 95.8	110.7 ± 48.6	< 0.001
Triglycerides at 2 h during MMT (mg/dL)	298.6 ± 128.4	132.1 ± 54.2	< 0.001
HDL-cholesterol (mg/dL)	42.4 ± 5.2	58.2 ± 13.1	< 0.001
LDL-cholesterol (mg/dL)	147.2 ± 26.5	96.2 ± 19.2	< 0.001
Fasting plasma glucose (mg/dL)	173.8 ± 63.9	92.0 ± 7.6	< 0.001
Postprandial 2 h glucose (mg/dL)	282.0 ± 97.1	103.2 ± 19.9	< 0.001
HbA1c (%)	8.3 ± 2.0	5.3 ± 0.2	< 0.001
Fasting plasma insulin (μIU/L)	10.3 ± 4.9	8.2 ± 3.0	0.097
HOMA-IR	4.3 ± 2.2	1.9 ± 0.7	< 0.001
HOMA-β	44.8 ± 27.4	104.0 ± 36.9	< 0.001
AST (IU/mL)	25.3 ± 11.1	25.9 ± 22.2	0.915
ALT (IU/mL)	32.3 ± 22.4	19.4 ± 11.9	0.029
Creatinine (mg/mL)	0.81 ± 0.18	0.78 ± 0.15	0.489
hsCRP (mg/dL)^a^	0.47 ± 1.40	0.07 ± 0.06	0.003
ADMA (mmol/L)	432.0 ± 48.7	374.5 ± 63.3	0.003
ADMA at 2 h during MMT (mmol/L)	458.3 ± 42.2	383.5 ± 63.4	< 0.001
PON-1 (μg/mL)	11.9 ± 2.2	13.5 ± 2.9	0.048
PON-1 at 2 h during MMT (μg/mL)	10.6 ± 1.4	13.8 ± 4.3	0.003
Microvascular reactivity using laser Doppler flowmetry			
Increase after ischemic challenge (%)	335.3 ± 123.4	579.3 ± 261.3	0.001

*DM* diabetes mellitus, *BMI* body mass index, *MMT* mixed-meal test, *HDL* high-density lipoprotein, *LDL* low-density lipoprotein, *HOMA-IR* homeostasis model assessment of insulin resistance, *HOMA-β* homeostasis model assessment of β-cell function, *AST* aspartate aminotransferase, *ALT* alanine aminotransferase, *hsCRP* high sensitivity C-reactive protein, *PON-1* paraoxonase 1, *ADMA* asymmetric dimethylarginine

^a^Log-transformed value was used for analysis

As expected, the patients had higher fasting levels of glucose, insulin, and HbA1c than the controls. Accordingly, HOMA-IR was greater and HOMA-β was lower in the patients than in the controls. Patient participants also had significantly higher levels of fasting total cholesterol, triglycerides, LDL-cholesterol, and hsCRP, and lower levels of HDL-cholesterol. Fasting and 2 h postprandial levels of ADMA were significantly higher in the patients than in the controls. By contrast, fasting and 2 h postprandial levels of PON-1 were significantly lower in the patients than in the controls. Postocclusive microvascular reactivity was significantly lower in the patients than in the controls (*P* < 0.05), suggesting altered endothelial function.

### Changes in biochemical parameters, including ADMA and PON-1, and microcirculation after rosuvastatin treatment

All 20 study participants completed 12 weeks of treatment with rosuvastatin. As shown in Table 2, BMI, glycemic indices, HOMA-IR, and HOMA-β did not change after 12 weeks of treatment with 20 mg rosuvastatin. Total cholesterol, triglycerides, and LDL-cholesterol levels decreased significantly, while HDL-cholesterol increased significantly in response to rosuvastatin treatment. Circulating concentrations of hsCRP also decreased significantly after rosuvastatin treatment. The degree of postocclusive reactive hyperemia increased by 20.1% (from 335.3 ± 123.4 to 402.7 ± 133.4%) after same duration of treatment (Table 2), suggesting altered microcirculation.

**Table 2:** Changes in biochemical parameters and microcirculation from baseline to 12 weeks after the administration of rosuvastatin (20 mg daily) in patients with type 2 diabetes and dyslipidemia

Parameters	Baseline	At 12 weeks	P
BMI (kg/m^2^)	24.6 ± 2.8	24.8 ± 2.7	0.114
Total cholesterol (mg/dL)	233.4 ± 36.5	132.7 ± 28.7	< 0.001
Triglycerides (mg/dL)	230.5 ± 95.8	151.1 ± 69.6	0.002
Triglycerides at 2 h during MMT (mg/dL)	298.6 ± 128.4	186.3 ± 78.0	< 0.001
HDL-cholesterol (mg/dL)	42.4 ± 5.2	44.7 ± 6.2	0.041
LDL-cholesterol (mg/dL)	147.2 ± 26.5	68.3 ± 24.5	< 0.001
Fasting plasma glucose (mg/dL)	173.8 ± 63.9	152.4 ± 60.9	0.081
Postprandial 2 h glucose (mg/dL)	282.0 ± 97.1	264.2 ± 102.7	0.489
HbA1c (%)	8.3 ± 2.0	8.0 ± 1.8	0.559
Fasting plasma insulin (μIU/L)	10.3 ± 4.9	14.1 ± 17.4	0.282
HOMA-IR	4.3 ± 2.2	5.1 ± 5.9	0.486
HOMA-β	44.8 ± 27.4	80.0 ± 98.6	0.110
AST (IU/mL)	25.3 ± 11.1	30.8 ± 19.1	0.100
ALT (IU/mL)	32.3 ± 22.4	35.8 ± 21.7	0.348
Creatinine (mg/mL)	0.81 ± 0.18	0.80 ± 0.10	0.713
hsCRP (mg/dL)^b^	0.47 ± 1.40	0.10 ± 0.09	0.014
ADMA (mmol/L)	432.0 ± 48.7	415.3 ± 51.6	0.040
ADMA at 2 h during MMT (mmol/L)	458.3 ± 42.2	419.0 ± 49.4	< 0.001
PON-1 (μg/mL)	11.9 ± 2.2	12.6 ± 2.5	0.066
PON-1 at 2 h during MMT (μg/mL)	10.6 ± 1.4	12.5 ± 2.2	0.001
Microvascular reactivity using laser Doppler flowmetry			
Increase after ischemic challenge (%)	335.3 ± 123.4	402.7 ± 133.4	0.006

*MMT* mixed-meal test, *PON-1* paraoxonase 1, *ADMA* asymmetric dimethylarginine

Fasting ADMA levels decreased by 3.87% and fasting PON-1 levels increased by 5.88% after treatment with rosuvastatin for 12 weeks (*P* = 0.040 and *P* = 0.066, respectively). Levels of ADMA 2 h postprandially decreased by 8.58% and those of PON-1 increased by 17.92% (both *P* < 0.01). Thus, the changes in fasting levels of both markers were modest compared with the changes in 2 h postprandial levels.

As shown in Fig. 1, the decrement in postprandial ADMA levels was significantly greater than the decrement in fasting ADMA levels (*P* = 0.025). The increment in postprandial PON-1 levels was significantly greater than the increment in fasting PON-1 levels (*P* = 0.041).

**Fig. 1:** Comparison of changes in ADMA and PON-1 levels under fasting conditions and 2 h postprandially (PP2) during a mixed-meal test at baseline and after 12 weeks of treatment with 20 mg rosuvastatin. *P indicates a comparison of changes in fasting levels and 2 h postprandial levels using an independent *t* test. *ADMA* asymmetric dimethylarginine, *PON-1* Paraoxonase-1

Correlations between changes in ADMA or PON-1 and changes in microvascular reactivity were analyzed to determine whether they were directly associated. As shown in Fig. 2b, d, the changes in 2 h postprandial levels of ADMA and PON-1 after a mixed-meal test were correlated with changes in microvascular reactivity significantly. By contrast, there was no significant correlation between changes in fasting levels of ADMA or PON-1 and changes in microvascular reactivity (Fig. 2a, c).

**Fig. 2:** Correlation between changes in fasting and 2 h postprandial (PP2) levels of ADMA (**a**, **b**) and PON-1 (**c**, **d**) during a mixed-meal test, and changes in microvascular reactivity (microcirculation). *ADMA* asymmetric dimethylarginine, *PON-1* Paraoxonase-1

## Discussion

In the present study, circulating levels of ADMA and hsCRP were significantly higher and levels of PON-1 were significantly lower in the patients than in the age- and BMI-matched healthy controls. In the intervention study, treatment with 20 mg rosuvastatin for 12 weeks improved postocclusive microvascular reactivity in the upper extremities, and increased PON-1 levels and decreased ADMA levels both under fasting conditions and 2 h postprandially. In particularly, changes in postprandial levels of PON-1 and ADMA after rosuvastatin treatment were significantly associated with improvement in microvascular reactivity.

Endothelial function impairment is considered a pathophysiological starting point in the initiation and progression of atherosclerotic vascular diseases [24]. Commonly, endothelial dysfunction is caused by endothelial damage and leads to subsequent events such as vascular stenosis, platelet aggregation, inflammation, and oxidative stress. Ultimately, this series of processes leads to the rupture of atheromatous plaques, resulting in an acute coronary syndrome [25].

Unfortunately, it is difficult to assess endothelial function at an early stage in vivo, despite much effort to do so. Flow-mediated dilation is used for this purpose, but it is somewhat examiner-dependent and not always available. In our study, we assessed postocclusive microvascular reactivity to detect early endothelial dysfunction using laser Doppler flowmetry. Microvascular reactivity was used as an early marker of endothelial dysfunction in women with gestational diabetes [17]. Microvascular circulatory function was assessed using laser Doppler flowmetry in patients with T2D [26].

Among the many biomarkers related to vascular health, ADMA and PON-1 reflect endothelial dysfunction and are known as early markers for cardiovascular events. High ADMA levels are associated with increases in cardiovascular events such as myocardial infarction, percutaneous coronary intervention, coronary-artery bypass graft, stroke, and carotid revascularization in patients with T2D [27]. Elevated levels of ADMA are independently associated with an increased risk of poor cardiovascular outcomes in T2D patients with coronary artery disease (CAD) [28]. Thus, clinical studies have proven a significant association between high ADMA levels and worse cardiovascular outcomes. A recent study reported that the circulating levels of ADMA were not altered after 12 weeks of treatment with trelagliptin, a dipeptidyl peptidase-4 inhibitor [29]. Additional studies are needed to corroborate the clinical value of ADMA as a cardiovascular biomarker.

The evidence on the effects of statin treatment on ADMA levels is inconsistent. A meta-analysis reported that hydrophilic statins such as rosuvastatin, pravastatin, and fluvastatin decrease ADMA levels, while hydrophobic statins such as atorvastatin or simvastatin do not alter ADMA levels [30]. However, there is no study that has investigated whether changes in ADMA levels after statin treatment are associated with an improvement in microcirculation.

In the present study, ADMA levels decreased after treatment with 20 mg rosuvastatin, and the decrement in ADMA levels during a mixed-meal test was associated with improved microvascular reactivity. Two potential mechanisms underlying this finding can be suggested. First, statins upregulate both proprotein convertase subtilisin/kexin type 9 mRNA levels and LDL receptor protein via activation of sterol-regulatory-element-binding protein-2, an important activator of dimethylarginine dimethylaminohydrolase (DDAH) transcription and activity [31]. Second, statins inhibit ADMA-induced inflammation, which is modulated by a mitogen-activated protein kinase (MAPK) pathway in endothelial cells [32]. Rosuvastatin preserves endothelial function through stimulation of vascular endothelial NO [33]. Taken together, these studies suggest that statin therapy might decrease ADMA levels through decreasing inflammation aggravated by MAPK pathways and/or activation of decreased activity of DDAH, which is linked to endothelial dysfunction.

PON-1 has drawn attention because of its association with cardiovascular and metabolic disorders [14]. A case–control study suggests that lower PON-1 activity and higher oxidized LDL levels are independently associated with CAD [34]. PON-1 activity is associated with HDL function, such as diminishing malondialdehyde formation [35]. Moreover, PON-1 inactivation leads to greater activation of protein kinase C-β, which is closely linked to endothelial dysfunction [36], and decreased phosphorylation of eNOS-Ser1177. This process blunts NO production, aggravates monocyte–endothelial cell adhesion, and impairs the endothelial repair system. These findings suggest a potential mechanistic link between decreased PON-1 activity and endothelial function. Furthermore, HDL fails to stimulate NO production or to antagonize endothelial inflammatory activation from *Pon1* ^−*/*−^ mice [35]. These findings indicate that PON-1 has an important impact on endothelial function, which is consistent with the results of our present study and those of others [37].

In addition to their lipid-lowering effect, several other mechanisms could be inferred to explain the improvement in microvascular function observed after treatment with statins, particularly rosuvastatin. Improvement in endothelial function after rosuvastatin treatment has been demonstrated in studies performed in animals and patients with heart failure [38, 39]. In an in vitro study, rosuvastatin treatment also suppressed the expression of the alkaline phosphatase mRNA, a proposed mechanism for vascular calcification [40], leading to impaired vascular reactivity. Alleviation in inflammatory processes by statin treatment was proven in cell studies [41, 42]. Decrease in inflammatory markers by rosuvastatin treatment was also found in clinical studies [43, 44], and was associated with mitigation of the progression of atherosclerosis and reduction of cardiovascular events. In most cases, these changes were not associated directly with changes in lipid levels, which indicates that rosuvastatin has multifactorial effects on vascular function beyond its direct lipid-lowering action. Along these lines, the serum levels of ADMA, a novel biomarker reflecting endothelial dysfunction, and PON-1, a specific enzyme with antioxidant and antiatherosclerotic properties, were modulated in a positive direction by rosuvastatin treatment, especially after fat loading, in the present study (Fig. 2). These findings support the potential favorable effect of rosuvastatin on microvascular reactivity beyond its lipid-lowering effect.

Postprandial hyperlipidemia triggers the proatherosclerotic processes of endothelial cells and is more closely related to early endothelial dysfunction than are fasting levels [45]. In subjects with T2D, such postprandial hyperlipidemia is prominent, long lasting, and finally contributes to increased risks of atherosclerotic disease. The therapeutic roles of lipid-lowering agents, including statins and ezetimibe, which lower lipid levels and inhibit the inflammatory process, have been proven to be superior regarding postprandial status [46, 47]. Consistently, the effects of rosuvastatin in improving atherosclerotic biomarkers are stronger in postprandial conditions, and were closely correlated with the improvement of microvascular reactivity in the present study.

Our present study has several limitations. First, our study population comprised only a small number of relatively healthy patients with T2D and dyslipidemia. Second, the duration of treatment was short, so long-term effects could not be evaluated. Third, antidiabetic treatments in the present study were diverse, including drug-naïve, treatment with metformin, or a combination of metformin with sulfonylurea; this may affect ADMA or PON-1 levels. Nevertheless, these treatments were maintained throughout the study period.

Our present study also has several advantages. First, we assessed circulation in small vessels using laser Doppler flowmetry, which has been validated for assessing endothelial dysfunction [17, 18]. Second, a standardized mixed-meal was given to the study participants to measure postprandial levels of PON-1 and ADMA in a standardized fashion. The changes in postprandial levels of PON-1 and ADMA were associated with microcirculation in small vessels after rosuvastatin treatment.

In the present study, treatment with 20 mg rosuvastatin decreased hsCRP levels, which is consistent with the results of other studies [3]. HsCRP reflects low-grade inflammation and has links to future cardiovascular events through having a deleterious effect on endothelial integrity [48].

In conclusion, treatment with 20 mg rosuvastatin improved microvascular reactivity in patients who had both diabetes and dyslipidemia. The favorable changes observed in the levels of biomarkers, i.e., increased PON-1 and decreased ADMA levels, which are related to endothelial function, were significantly associated with an improvement in microvascular reactivity. Our present findings suggest that, in addition to the lipid-lowering effects of rosuvastatin treatment, improved circulation in small vessels may contribute to its positive outcomes on cardiovascular morbidity and mortality.

## Additional file

**Additional file 1: Table S1.** Amount and percentage* of nutritional components contained in 100 mL of a can of New Care.

## Abbreviations

T2D: type 2 diabetes
LDL: low-density lipoprotein
ADMA: asymmetric dimethylarginine
PON-1: paraoxonase-1
NO: nitric oxide
AST: aspartate aminotransferase
ALT: alanine aminotransferase
BMI: body mass index
HbA1c: glycated hemoglobin
HOMA-IR: homeostasis model assessment of insulin resistance
HOMA-β: homeostasis model assessment of β-cell function
hsCRP: high sensitivity C-reactive protein
CAD: coronary artery disease
HDL: high-density lipoprotein
MMT: mixed-meal test
SD: standard deviation
MAPK: mitogen-activated protein kinase
DDAH: dimethylarginine dimethylaminohydrolase
